RETRACTED

# Deletion of the scavenger receptor Scarb1 in myeloid cells does not affect bone mass

**DOI:** 10.1016/j.bone.2023.116702

**Published:** 2023-02-10

**Authors:** Michela Palmieri, Teenamol E. Joseph, Charles A. O'Brien, Horacio Gomez-Acevedo, Ha-Neui Kim, Stavros C. Manolagas, Elena Ambrogini

**Affiliations:** a Division of Endocrinology and Metabolism, Center for Osteoporosis and Metabolic Bone Diseases, the Center for Musculoskeletal Disease Research, University of Arkansas for Medical Sciences, Central Arkansas Veterans Healthcare System, Little Rock, AR, USA; b Department of Biomedical Informatics, University of Arkansas for Medical Sciences, Little Rock, AR, USA

**Keywords:** Scavenger receptor class B member 1 (SR-B1 or Scarb1), Macrophages, Osteoclasts, Oxidized phospholipids, Bone mass

## Abstract

The scavenger receptor class B member 1 (SR-B1 or Scarb1) is a glycosylated cell surface receptor for high density lipoproteins (HDL), oxidized low density lipoproteins (OxLDL), and phosphocholine-containing oxidized phospholipids (PC-OxPLs). Scarb1 is expressed in macrophages and has been shown to have both pro- and anti-atherogenic properties. It has been reported that global deletion of Scarb1 in mice leads to either high or low bone mass and that PC-OxPLs decrease osteoblastogenesis and increase osteoclastogenesis. PC-OxPLs decrease bone mass in 6-month-old mice and are critical pathogenetic factors in the bone loss caused by high fat diet or aging. We have investigated here whether Scarb1 expression in myeloid cells affects bone mass and whether PC-OxPLs exert their anti-osteogenic effects *via* activation of Scarb1 in macrophages. To this end, we generated mice with deletion of Scarb1 in LysM-Cre expressing cells and found that lack of Scarb1 did not affect bone mass *in vivo*. These results indicate that Scarb1 expression in cells of the myeloid/osteoclast lineage does not contribute to bone homeostasis. Based on this evidence, and earlier studies of ours showing that Scarb1 expression in osteoblasts does not affect bone mass, we conclude that Scarb1 is not an important mediator of the adverse effects on PC-OxPLs in osteoclasts or osteoblasts in 6-month-old mice.

## 1. Introduction

The scavenger receptor class B member 1 (SR-B1 or Scarb1) is a glycosylated cell surface receptor expressed in many tissues and cell types. Scarb1 is primarily a receptor for high density lipoproteins (HDL) and mediates the uptake of cholesteryl esters from HDL, as well as the efflux of cellular cholesterol to HDL [1,2]. Importantly, Scarb1 binds to oxidized low density lipoproteins (OxLDL) and phosphocholine-containing oxidized phospholipids (PC-OxPLs) [3-5].

RETRACTED

PC-OxPLs are pro-inflammatory adducts that are neutralized by the natural antibody E06 IgM.

Male and female transgenic mice expressing a single chain (scFv) form of the antigen-binding domain of E06 IgM (E06-scFv) have increased trabecular and cortical bone mass at 6 months of age [6,7], and are protected from the bone loss caused by a high fat diet or aging [6,8]. This evidence indicates that PC-OxPLs affect bone metabolism under both physiological and pathological conditions. E06-scFv increases osteoblast number and bone formation rate and decreases osteoclast number in vertebral bone throughout life [7,8]. However, the mechanisms by which PC-OxPLs affect bone mass remain unclear. We had hypothesized that PC-OxPLs may affect bone mass by binding to Scarb1 in osteoblasts. Mice with germline deletion of Scarb1 (Scarb1 KO) have increased osteoblast number, bone formation rate, and high bone mass, similar to E06-scFv transgenic mice [9-11]. Moreover, osteoblasts from Scarb1 KO mice are protected from the pro-apoptotic and anti-differentiating effects of OxLDL in culture [7]. However, in our previous work, we found that deletion of Scarb1 in osteoblast lineage cells (targeted by Osx1-Cre) did not affect bone mass or architecture, suggesting that Scarb1 does not mediate the deleterious effects of PC-OxPLs on osteoblasts [12]. In the present study we have tested the alternative hypothesis that PC-OxPLs may exert their anti-osteogenic effects *via* activation of Scarb1 in macrophages, possibly leading to increased production anti-osteoblastogenic cytokines, such as TNF-α [13]. To this end, we deleted Scarb1 specifically in myeloid cells using LysM-Cre mice. We report that lack of Scarb1 in myeloid progenitors and their descendants does not alter bone mass *in vivo.* We conclude that Scarb1 expression in either osteoblasts or osteoclasts is not involved in bone homeostasis and, therefore, Scarb1 is not a major mediator of the deleterious effects of PC-OxPLs on bone.

## 2. Materials and methods

### 2.1. Animals

The mouse line harboring the Scarb1 conditional allele has been previously described [12,14]. To delete Scarb1 in the entire myeloid lineage, Scarb1 floxed mice were crossed with LysM-Cre mice, purchased from Jackson Laboratories (stock number 004781) [15]. All mice were in the C57BL/6 background.

To obtain experimental animals, a two-step breeding strategy was used. We crossed homozygous LysM-Cre transgenic mice with homozygous Scarb1 floxed mice (Scarb1^fl/fl^) to generate mice heterozygous for the Scarb1 (Scarb1^fl/+^) allele and the LysM-Cre allele. Those mice were then crossed with Scarb1^fl/+^ mice, to generate the control group of Scarb1^fl/fl^ mice and the experimental group, LysM-Cre;Scarb1^fl/fl^ mice. All mouse strains were fed a regular chow diet [Lab Diet 5 K67 Mouse/6F Diet (Lab Diet, St. Louis, MO, USA)]. Mice were group housed under specific pathogen-free conditions and maintained at a constant temperature of 23 °C, in a 12:12-h light-dark cycle; they had *ad libitum* access to diet and water.

RETRACTED

We genotyped offspring by PCR using the following primer sequences: Cre-Fwd: 5′-GCTAAACATGCTTCATCGTCGG-3′, Cre-Rev: 5′-GATCTCCGGTATTGAAACTCCAGC-3′, product size 650 bp; Scarb-WT-Fwd: 5′-AAAGAGGGCAGGTGCAGTAAGCGAAG-3′, Scarb-WT-Rev: 5′-TTTCAGTGACAGTGGGCTTCTCTGGG-3′, product size wild type 223 bp, heterozygous 223 and 346 bp; Scarb_tm1c distal loxp-Fwd: 5′ GCGCAACGCAATTAATGATAAC-3′, Scarb_tm1c distal loxp-Rev: GTCCAAGACTCCCTCCAAACGCACG-3′, product size floxed 222 bp.

### 2.2. Imaging

We used a PIXImus densitometer (GE Lunar) for dual-energy X-ray absorptiometry (DXA) measurements of bone mineral density (BMD) and percentages of lean and fat body mass, as previously described [7,16]. For these measurements, mice were sedated with 2 % isoflurane. The mean coefficient of variation was calculated using a proprietary phantom scanned at the beginning of each session for the duration of the study and was −0.46 % for BMD and −0.47 % for the percentage of body fat.

A micro-CT40 scanner from Scanco Medical (AG, Brüttisellen, Switzerland) was used to measure bone microarchitecture, as previously described [6,7]. For trabecular bone measurements, we used the fifth lumbar vertebra (L5) and the metaphysis of left femur, whereas cortical bone was measured at the left femoral diaphysis (midpoint of the bone length as determined in scout view). Prior to analysis, the bones were processed as previously described [7]. Briefly, L5 and the left femur were fixed using 10 % Millonig's Neutral Buffered Formalin with 5 % sucrose (Leica Biosystems Inc., Buffalo Grove, IL, USA). Bones were kept in 100 % ethanol until analysis. While performing these studies, the mean coefficient of variation of the micro-CT phantom was monitored weekly and was 0.147 %.

### 2.3. Histomorphometry

L1-L3 vertebra were dissected, fixed in 10 % Millonig's neutral buffered formalin with 5 % sucrose, dehydrated with ethanol, and stored in 100 % ethanol until embedding in methyl methacrylate (Sigma-Aldrich, St Louis, MO, USA). To measure the static indices of osteoclast number and surface, five μm thick longitudinal sections of trabecular bone were stained for tartrate-resistant acid phosphatase (TRAP) with the Leukocyte Acid Phosphatase (TRAP) Kit from Sigma-Aldrich (cat number 387A). Briefly, deplasticized sections were stained with TRAP solution (a mixture of Fast Garnet GBC Base Solution, Sodium Nitrite Solution, Napthol AS-BI Phosphate Solution, Acetate Solution, Tartrate Solution) for 1 h and 45 min at 37C. Histomorphometric determinations were made at L3, in a blinded fashion using Osteomeasure version 7 V4.3.0.0 (OsteoMetrics Inc. Decatur, GA, USA) as previously described [6]. Histomorphometric data are reported using the nomenclature recommended by the American Society for Bone and Mineral Research [17].

RETRACTED

### 2.4. In vitro osteoclast formation

Total bone marrow cells were harvested from femurs and tibias of 6-month-old Scarb1^fl/fl^ and LysM-Cre;Scarb1^fl/fl^ mice. After removing red blood cells with ACK buffer (0.1 mM EDTA, 10 mM KHCO3 and 150 mM NH4Cl, pH 7.2–7.3), bone marrow cells were plated in 10 cm tissue culture plates with 10 ml α-MEM complete media (10 % fetal bovine serum, 100 U/ml penicillin, and 100 μg/ml streptomycin) supplemented with macrophage colony-stimulating factor (M-CSF; 30 ng/ml; cat. 216-MC, R&D Systems Minneapolis, MN). After 24 h of incubation, non-adherent cells were plated in Petri dishes (10 cm) and cultured with 10 ml α-MEM complete media supplemented with M-CSF (30 ng/ml) for 4 days. Those cells were used to culture macrophages and osteoclasts for analysis of mRNA and gDNA.

To obtain mRNA and genomic DNA, cells were then plated in 6-well plates at a density of 0.3 × 10^6^ cells/well with 1.5 ml of α-MEM complete media supplemented with 30 ng/ml M-CSF for 3 days to obtain macrophages and with 30 ng/ml M-CSF and 30 ng/ml RANKL (RANKL cat. 462-TEC, R&D Systems, Minneapolis, MN, USA) for 3 days to obtain osteoclasts.

### 2.5. Genomic DNA extraction and gene expression analysis

To obtain genomic DNA from macrophages and osteoclasts, cells were digested with proteinase K (Cat. P5850, Sigma-Aldrich) in a buffer (0.67 mg/ml in 30 mM TRIS, pH 8.0, 200 mM NaCl, 10 mM EDTA, and 1 % SDS) at 55 °C overnight. The right kidney was harvested, cut in 3–4 pieces, frozen in liquid nitrogen and digested with proteinase K as described above. Genomic DNA was purified by phenol/chloroform extraction and ethanol precipitation. A custom Taqman assay was obtained from Applied Biosystems to quantify the Scarb1 deletion efficiency in genomic DNA: Fwd 5′-GCACGTGTGCTTCATACAAATAGG-3′; Rev. 5′-ACTCACACTAGCACAGACATCTCTA-3′; probe 5′-TCTGGCCCTAGCACTCT-3′. The relative amount of genomic DNA was calculated with the ΔCt method using an assay for the transferrin receptor gene (Tfrc) as a control [18].

### 2.6. mRNA extraction and gene expression analysis

Total RNA was extracted from macrophages, osteoclasts, and vertebral bone (L6) with Trizol (Thermo Fisher Scientific, cat. 15,596,026, Waltham, MA, USA) and purified with Direct-zol RNA Miniprep kits (cat. R2050, Zymo Research, Irvine, CA, USA) according to manufacturer's instructions. RNA quantity and 260/280 ratio were determined using a NanoDrop instrument (Thermo Fisher Scientific), and its integrity was verified by resolution on 1 % agarose gels. Complementary DNA (cDNA) was reverse transcribed from 0.5 μg of total RNA using the High-Capacity cDNA Reverse Transcription kit (cat. 4,368,813, Applied Biosystems, Foster City, CA, USA) according to manufacturer's instructions. PCR was performed using a custom TaqMan Gene Expression Assays manufactured by Applied Biosystems, as listed in Supplementary Table 1. Transcript levels were calculated by normalizing to the reference mRNA Mitochondrial Ribosomal Protein S2 (MRPS2) using the ΔCt method [18].

RETRACTED

### 2.7. Bone remodeling markers

Bone remodeling markers, N-terminal propeptide (P1NP) and tartrate-resistant acid phosphatase (TRAP) were measured with an ELISA kit [cat. AC-33F1 for P1NP and cat SB-TR103 for TRAP, Immunodiagnostic Systems, Boldon Colliery, UK] according to manufacturer's instructions.

### 2.8. Statistics

No experimentally derived data were excluded. In Fig. 4B and D, the femoral length could not be measured in 1 male Scarb1^fl/fl^ mouse and in 3 female and 2 male LysM-Cre;Scarb1^fl/fl^ mice because the head of the femur was damaged during the harvest. Each figure legend includes the number of mice or samples used in each experiment. Single data points are shown in Figs. 1, 3-5 with mean ± standard deviation. In Fig. 2 the data are shown as mean ± standard deviation.

Statistical analyses were performed using GraphPad Prism (versions 7.0.4 and 8.0.1). Statistical analysis for the data shown in Fig. 2 was performed using R (version 3.6). Group mean values were compared by Student's two-tailed *t*-test or ANOVA repeated measures as appropriate.

For the *in vivo* studies, the sample size was adequate to detect a difference of 1.2 standard deviations at a power of 0.8, and *p* < 0.05 [13]. For *in vitro* experiments, the number of replicates was sufficient to provide confidence in the measurements. All data were collected and analyzed by personnel blinded to the identity of the samples.

### 2.9. Study approval

This study was carried out in strict accordance with the recommendations in the Guide for the Care and Use of Laboratory Animals of the National Institutes of Health. The animal protocols were approved by the Institutional Animal Care and Use Committees of the Central Arkansas Veterans Healthcare System (IACUC protocol # 1400199). Euthanasia was performed by CO2 inhalation from a compressed gas tank and death was verified by lack of respiration and cervical dislocation as previously reported.

RETRACTED

## 3. Results

### 3.1. Scarb1 was successfully deleted in LysM-Cre-targeted cells

To delete Scarb1 in monocytes and macrophages, we crossed mice Scarb1^fl/fl^ mice [12] with transgenic mice expressing Cre recombinase under the control of LysM-Cre regulatory elements (LysM-Cre mice) [15]. The phenotype of LysM-Cre;Scarb1^fl/fl^ mice was compared with Scarb1^fl/fl^ littermate controls. We first quantified deletion of the Scarb1 gene in bone marrow-derived macrophages and osteoclasts from 6-month-old female and male mice. We found that the levels of Scarb1 floxed exons were 74.2 % and 87.5 % lower in macrophages and osteoclasts derived from LysM-Cre;Scarb1^fl/fl^ female mice and 84.3 % and 79.9 % lower in macrophages and osteoclasts derived from LysM-Cre;Scarb1^fl/fl^ male mice as compared with Scarb1^fl/fl^ littermate controls, confirming deletion of the gene (Fig. 1A, C). There were no changes in Scarb1 DNA levels in the kidney, confirming the specificity of the deletion (Fig. 1A, C). We also quantified the effectiveness of our deletion strategy for Scarb1 at the mRNA level and found that Scarb1 RNA abundance was 63.6 % and 84.2 % lower in macrophages and osteoclasts derived from LysM-Cre;Scarb1^fl/fl^ female mice (Fig. 1B), and 76.6 % and 73.9 % lower in macrophages and osteoclasts derived from LysM-Cre;Scarb1^fl/fl^ male mice, as compared with Scarb1^fl/fl^ controls (Fig. 1D). This level of deletion is comparable to the one obtained in other experiments in which we used LysM-Cre mice to delete other genes in the myeloid/osteoclast lineage [19-21].

### 3.2. Deletion of Scarb1 in LysM-Cre-targeted cells does not affect body weight, fat mass, or bone mass

We then analyzed the skeletal phenotype of Scarb1^fl/fl^ and LysM-Cre;Scarb1^fl/fl^ mice. All mice gained weight throughout the observational period and there were no differences between the genotypes (Fig. 2A). There was also no difference in fat mass and lean mass at 2, 4 and 6 months of age in female and male mice (Fig. 2A, B). Bone mineral density measured by DXA at the same time points showed no difference between genotypes in either female or male mice (Fig. 2A, B).

Micro-CT analysis of 6-month-old mice revealed no differences between genotypes in trabecular bone in the vertebra or the femur of either sex (Fig. 3).

We also did not detect any change in cortical thickness, total area, medullary area, or femoral length in either female or male mice (Fig. 4). Overall, these results demonstrate that deletion of Scarb1 in cells of the myeloid lineage does not alter bone mass in growing or adult mice.

Consistent with the lack of changes in bone mass measured by BMD or micro-CT, there was no difference in serum P1NP, a marker of bone formation, or serum TRAP, a marker of bone resorption, in either female or male mice (Fig. 5 A). Quantification of mRNA encoding osteoclast markers in vertebral bone showed a decrease in cathepsin K in female mice but unchanged levels of Acp5, which encodes TRAP, and Igtb3, which encodes a beta integrin subunit, between genotypes (Fig. 5 B). Deletion of Scarb1 in myeloid cells did not change the osteoclast number or surface in vertebral trabecular bone (Fig. 5 C). These results confirm that deletion of Scarb1 in cells of the myeloid/osteoclast lineage does not affect bone mass or architecture *in vivo.*

RETRACTED

## 4. Discussion

Scarb1 is a high affinity receptor for high density lipoproteins (HDL) and facilitates the selective uptake of cholesteryl esters from HDL into the liver. In addition to being a receptor for HDL, Scarb1 has been implicated in the plasma clearance of low-density lipoproteins (LDL), very low-density lipoproteins (VLDL) and lipoprotein (a) [Lp(a)]; the latter being the major carrier for oxidized phospholipids [3,22,23]. Scarb1 binds to OxLDL and the phosphocholine moiety of oxidized phospholipids (PC-OxPLs) [4,5,24].

PC-OxPLs have deleterious effects on bone [6-8]. Moreover, we have shown earlier that transgenic mice overexpressing E06-scFv – the monomeric form of the antigen recognition portion of E06 IgM, a natural antibody that blocks PC-OxPL – have increased bone mass at 6 months of age and are protected from the bone loss caused by high fat diet or aging [6-8]. We have also shown previously that the E06-scFv transgene increases osteoblast number and bone formation rate at both trabecular and cortical sites, reduces osteoblast apoptosis *in vivo,* and decreases osteoclasts in trabecular bone [7,8]. Consistent with this, E06 IgM prevents the negative effects of OxLDL on the proliferation, differentiation, and survival of osteoblastic cells *in vitro.*

The mechanisms by which E06-scFv increases osteoblast number and function remains unclear. We had initially hypothesized that Scarb1 was an essential mediator of the pro-apoptotic effects of PC-OxPLs on osteoblasts [4]. However, our previous work showed that deletion of Scarb1 in osteoblastic lineage cells did not affect bone mass or architecture, demonstrating that Scarb1 does not mediate the deleterious effects of PC-OxPLs on osteoblasts or bone [12]. Therefore we tested the alternative possibility that PC-OxPLs may exert their anti-osteogenic effects *via* activation of Scarb1 in macrophages [13].

The role of Scarb1 in macrophages has been extensively studied in mouse models of atherosclerosis where it has been found to be both proatherogenic and anti-atherogenic [25]. Whereas earlier reports indicate that deletion of Scarb1 reduced the development of atherosclerosis [26], a recent study showed that deletion of this receptor in monocytes and macrophages worsened the extension of atherosclerotic lesions at earlier stages [27]. Specifically, Scarb1 deficiency in LysM-Cre expressing cells increased atherosclerosis by increasing the expression of the apoptosis inhibitor of macrophages (AIM) protein and consequently reducing macrophage apoptosis. Since macrophage apoptosis is associated with attenuation of early atherogenesis, this study suggests that decreased apoptosis is responsible for the increased accumulation of macrophages in the atherosclerotic plaque and expansion of the lesions. In more advanced atherosclerotic lesions Scarb1 present in macrophages binds and mediates the removal of apoptotic cells by efferocytosis; the absence of Scarb1, therefore, increases the numbers of apoptotic cells that did not get removed and increases the necrosis of the atherosclerotic plaques [28]. Moreover, Scarb1 expression in macrophages induces expression of transcription factor EB (TFEB), a master regulator of autophagy, which limits the necrosis and increases stability of atherosclerotic plaques; deletion of Scarb1, therefore, impairs autophagy and worsens the atherosclerosis at later stages [29]. Heretofore, the role of Scarb1 in macrophages has not been studied in bone.

RETRACTED

Earlier attempts to determine the bone phenotype of mice with global deletion of Scarb1 (Scarb1 KO) have produced conflicting results. Martineu et al. reported that Scarb1 KO mice have increased trabecular bone at 2 and 4 months of age and this was associated with increased osteoblast surface, mineralized surface, and bone formation rate with no changes in osteoclasts parameters [9-11]. In contrast, Tourkova et al. showed that Scarb1 KO mice have low bone mass at 16 weeks of age with low bone formation and decreased osteoclastogenesis compared to WT mice, suggesting that Scarb1 is required for osteoblast and osteoclast differentiation [30].

The results presented herein show that deletion of Scarb1 in cell of the myeloid/osteoclast lineage does not affect bone mass in either female or male mice. This evidence indicates that Scarb1 expression in macrophages and osteoclasts does not play a major role in skeletal homeostasis. Scarb1, therefore, there may not be a major mediator of the deleterious effects of PC-OxPLs on bone homeostasis. PC-OxPLs bind to other scavenger receptors, such as CD36, and toll-like receptors, such as TLR2, 4 and 6 which may mediate the deleterious effects in bone and compensate for the lack of Scarb1 [4]. Our previous work has indicated that PC-OxPLs decreases Wnt signaling, and this decrease may mediate the negative effects of PC-OxPLs in bone [8]. Thus, identification of the mechanisms by which PC-OxPLs affect bone homeostasis will require further investigation.

RETRACTED

An important limitation of this study is that we did not challenge the mice with high fat diet or high cholesterol diet. It remains possible that Scarb1 in myeloid progenitors may play a role in inflammatory conditions with higher levels of oxidized phospholipids. This possibility will be pursued in future studies.

## Supplementary Material

Suppl. Table 1

## Figures and Tables

**Fig. 1.** Scarb1 gene was effectively deleted in LysM-Cre targeted cells. (A) Quantitative PCR (qPCR) of loxP-flanked genomic DNA isolated from macrophages, osteoclasts, and right kidney obtained from 6-month-old female mice. Macrophages and osteoclasts were cultured from bone marrow cells as described in the methods section [for macrophages and osteoclasts Scarb1^fl/fl^ (*n* = 2), LysM-Cre;Scarb1^fl/fl^ (*n* = 6), six replicates of pooled cultures; for kidney Scarb1^fl/fl^ (*n* = 10), LysM-Cre;Scarb1^fl/fl^ (*n* = 18)]. (B) Scarb1 expression quantified by RT-PCR in the same cells as in (A). (C) qPCR of loxP-flanked genomic DNA isolated from macrophages and osteoclasts obtained from 6-month-old male mice cultured as in (A) and genomic DNA isolated from right kidney from 6-month-old male mice; [for macrophages and osteoclasts Scarb1^fl/fl^ (n = 2), LysM-Cre;Scarb1^fl/fl^ (n = 2), six replicates of pooled cultures; for kidney Scarb1^fl/fl^ (n = 10), LysM-Cre;Scarb1^fl/fl^ (*n* = 15)]. (D) Scarb1 expression was quantified by RT-PCR of cells cultured as in (C). Transcripts were normalized to the reference gene MRPS2. Bar and whiskers are the mean ± standard deviation (s.d.) and *p* values were calculated using 2-tailed unpaired *t*-tests.

**Fig. 2.** Deletion of Scarb1 in LysM-Cre-targeted cells does not affect body weight, fat mass, lean mass, or BMD in either sex. (A) Body weight, fat mass, lean mass, and BMD measurements at the indicated sites at 2, 4 and 6 months of age in female mice [Scarb1^fl/fl^ *n* = 10; LysM-Cre;Scarb1^fl/fl^ *n* = 18]. (B) Weight, fat mass, lean mass, and BMD measurements at 2, 4 and 6 months of age in male mice [Scarb1^fl/fl^ *n* = 10; LysM-Cre;Scarb1^fl/fl^ *n* = 15]. Data are shown as mean and standard deviation. Adjusted *p* values, calculated by repeated measures using two-way ANOVA are shown. BMD: Bone mineral density.

**Fig. 3.** Deletion of Scarb1 using LysM-Cre does not affect trabecular bone in either sex. Micro-CT determination of trabecular bone architecture in (A) vertebral and femoral metaphyseal bone of 6-month-old female mice [Scarb1^fl/fl^ *n* = 10; LysM-Cre;Scarb1^fl/fl^ *n* = 18] and in (B) vertebral and femoral metaphyseal bone of 6-month-old male mice [Scarb1^fl/fl^ *n* = 10; LysM-Cre;Scarb1^fl/fl^ *n* = 15]. Bar and whiskers are the mean ± s.d. and *p* values were calculated using 2-tailed unpaired *t*-tests.

RETRACTED

**Fig. 4.** Deletion of Scarb1 using LysM-Cre does not affect cortical bone in female or male mice. (A, C) Micro-CT determination of cortical bone in 6-month-old female [Scarb1^fl/fl^ *n* = 10; LysM-Cre;Scarb1^fl/fl^ *n* = 18] and male mice [Scarb1^fl/fl^ n = 10; LysM-Cre;Scarb1^fl/fl^ *n* = 15]. (B, D) Femoral length in female [Scarb1^fl/fl^ n = 10; LysM-Cre;Scarb1^fl/fl^ n = 15] and male mice [Scarb1^fl/fl^ *n* = 9; LysM-Cre;Scarb1^fl/fl^ *n* = 13]. Bar and whiskers are the mean ± s.d. and *p* values were calculated with 2-tailed unpaired *t*-tests.

**Fig. 5.** Deletion of Scarb1 using LysM-Cre does not affect osteoclast number *in vivo*. (A) Measurement of bone remodeling markers in the serum of 6-month-old female and male mice [Scarb1^fl/fl^ *n* = 10; LysM-Cre;Scarb1^fl/fl^ n = 10], P1NP, N-terminal propeptide; TRAP, Tartrate-resistant acid phosphatase. (B, C) The expression of osteoclasts marker genes TRAP (Acp5), CTSK, and Igtb3 was quantified by RT-PCR in vertebral bone (L6) of 6-month-old female and male mice [Scarb1^fl/fl^ n = 10; LysM-Cre;Scarb1^fl/fl^ n = 10]. Transcripts were normalized to the reference gene transcript MRPS2. (D) Histomorphometric measurements of vertebral trabecular bone surface (L3); [Scarb1^fl/fl^ n = 10; LysM-Cre;Scarb1^fl/fl^ n = 10]. Bar and whiskers are the mean ± s.d. and *p* values were calculated using 2-tailed unpaired *t*-tests. CTSK: Cathepsin K; Igtb3: Integrin β3; N.Oc, osteoclast number; B.Pm, bone perimeter; Oc.S, osteoclast surface; BS, bone surface.

## Data Availability

The data sets generated and/or analyzed during the current study are available from the corresponding author upon reasonable request.
